The article "Canine Morbillivirus from Colombian Lineage Exhibits In Silico and In Vitro Potential to Infect Human Cells" was retracted in 2022. Reasons: contaminated cell lines or tissues; errors in the data; errors in the analysis; errors in the results or conclusions.

# Canine Morbillivirus from Colombian Lineage Exhibits In Silico and In Vitro Potential to Infect Human Cells

**DOI:** 10.3390/pathogens10091199

**Published:** 2021-09-15

**Authors:** Santiago Rendon-Marin, Carolina Quintero-Gil, Diego Guerra, Carlos Muskus, Julian Ruiz-Saenz

**Affiliations:** 1 Grupo de Investigación en Ciencias Animales—GRICA, Facultad de Medicina Veterinaria y Zootecnia, Universidad Cooperativa de Colombia, sede Bucaramanga, 680002 Bucaramanga, Colombia; santiago.rendonm@udea.edu.co (S.R.-M.); dcaro63@gmail.com (C.Q.-G.); 2 Programa para el Estudio y Control de Enfermedades Tropicales—PECET, Facultad de Medicina, Universidad de Antioquia, 050010 Medellín, Colombia; diegoguerraar@gmail.com (D.G.); carlos.muskus@udea.edu.co (C.M.)

**Keywords:** canine distemper, cellular receptor, inter-species transmission, Nectin-4, SLAM molecule

## Abstract

*Canine morbillivirus* (CDV) is a viral agent that infects domestic dogs and a vast array of wildlife species. It belongs to the *Paramyxoviridae* family, genus Morbillivirus, which is shared with the Measles virus (MeV). Both viruses employ orthologous cellular receptors, SLAM in mononuclear cells and Nectin-4 in epithelial cells, to enter the cells. Although CDV and MeV hemagglutinin (H) have similar functions in viral pathogenesis and cell tropism, the potential interaction of CDV-H protein with human cellular receptors is still uncertain. Considering that CDV is classified as a multi-host pathogen, the potential risk of CDV transmission to humans has not been fully discarded. In this study, we aimed to evaluate both in silico and in vitro, whether there is a cross-species transmission potential from CDV to humans. To accomplish this, the CDV-H protein belonging to the Colombian lineage was modelled. After model validations, molecular docking and molecular dynamics simulations were carried out between Colombian CDV-H protein and canine and human cellular receptors to determine different aspects of the protein–protein interactions. Moreover, cell lines expressing orthologous cellular receptors, with both reference and wild-type CDV strains, were conducted to determine the CDV cross-species transmission potential from an in vitro model. This in silico and in vitro approach suggests the possibility that CDV interacts with ortholog human SLAM (hSLAM) and human Nectin-4 receptors to infect human cell lines, which could imply a potential cross-species transmission of CDV from dogs to humans.

## 1. Introduction

Canine morbillivirus, also called canine distemper virus (CDV), is a viral pathogen that can be transmitted to a wide range of wild and domestic animals, including domestic dogs, which are the primarily affected species [1]. CDV can affect more than 8 orders and 20 animal families, including the endangered Amur tigers (*Panthera tigris altaica*) and the vulnerable giant pandas (*Ailuropoda melanoleuca*); therefore, it has garnered special interest [2]. The viral infection produces an acute febrile disease, with respiratory, gastrointestinal, and neurological pathologies.

As a member of the *Paramyxoviridae* family, genus *Morbillivirus*, which also includes MeV, Rinderpest and Cetacean morbillivirus, it contains a single-stranded, negative sense RNA genome, which is organized linearly in six transcription units and codes for eight proteins [3,4]. Among those proteins, the CDV envelope contains the hemagglutinin (H) and the fusion (F) proteins, both essential to facilitate viral attachment and entrance into the host cell [5]. To accomplish viral recognition and entry, two cellular receptors have been identified, SLAM (signaling lymphocyte activation molecule or CD150) present in T cells, immature thymocytes, memory T cells, a proportion of B cells, activated monocytes, and dendritic cells [6] and the poliovirus receptor-like protein 4 (PVRL4), also known as Nectin-4, lying in the conjunctive junction of the epithelial cells [7]. SLAM has two extracellular domains, a V loop and a C2 loop, and Nectin-4 has three Ig-like ectodomains, a V region, two C2 domains, a transmembrane region, and a cytoplasmic tail. The V region from both cellular receptors is crucial to the interaction with CDV-H protein [8]. Nectin-4 has been considered as a conserved cellular receptor among diverse species [9]; however, SLAM is a non-conserved receptor [10], so its interaction with the CDV-H protein likely defines the host range of CDV [11]. CDV-H protein binding to the SLAM receptor is mediated by interaction of the H protein with 11 amino acid residues from the SLAM receptor with an exposed region of the CDV-H protein located between residues 500 and 550 [12].

The H protein is the CDV binding protein to the host cell surface and belongs to the transmembrane glycoprotein type II that comprises a small N-terminal cytoplasmic tail, a transmembrane domain, and a large C-terminal ectodomain [5]. The encoding gene for the H glycoprotein is estimated as the most variable among CDV lineages [13]. Based on the full sequence of the H gene from CDV strains isolated worldwide [14], to date, diverse genotypes have been described: America-1 (which includes almost all commercially available vaccine strains), America-2 to -5, Arctic-like, Rockborn-like, Asia-1 to -4, Africa-1 to -2, European Wildlife, Europe/South America-1, South America-2 and -3 and South/North America-4 [15,16,17,18,19,20,21,22,23,24,25,26]. The South American 3 lineage was previously described as circulating among domestic dog populations in Colombia [27]. This lineage exhibited differences in the amino acidic sequence in comparison to vaccine and wild-type strains circulating around the world [17]. However, the consequences of these amino acid changes to the 3D structure and the interaction with host cell receptors have not yet been investigated. In addition to initial viral binding to the host cell receptor, other factors may be affected by amino acid changes, including host immune system response and virus neutralization, but the effects remain unclear [28].

To understand protein–protein interactions, computational tools such as homology modelling, molecular docking and molecular dynamics have become useful alternatives, although the lack of crystallographic structures for the CDV-H proteins and canine cellular receptors has hindered these types of studies. Nevertheless, structural biology assays based on MeV H protein crystallography have demonstrated the interacting interfaces between this viral protein and the cellular receptors, both SLAM and Nectin-4. Considering that CDV has widely been accepted as a surrogate model of MeV, this MeV H protein information could be extrapolated to the CDV-H protein [29,30].

It is well known that CDV can infect non-human primates causing a devastating disease [31]; however, to date, there has been no evidence of CDV cross-species infection in humans, although CDV has been isolated in human cancer cell lines, including breast, lung, and prostate, which express the human Nectin-4 (hNectin-4) receptor in vitro. Hence, CDV binds efficiently to hNectin-4 to allow cellular uptake and infection. However, although CDV binds to canine SLAM (cSLAM) receptors efficiently in vitro, cellular infection has been unsuccessful using hSLAM receptors [32]. This fact could be explained through the small species-related variation in the Nectin-4 sequences between humans, mice, dogs, and other animal species, in comparison to the considerable variation in the SLAM sequence [9]. An interspecific study of SLAM receptors, employing recombinant SLAM proteins from different species including dogs and humans, as well as recombinant H proteins from MeV and CDV, demonstrated that there is a relatively strict tropism of CDV to cSLAM. However, some mutation sites on CDV-H could enable adaptation to hSLAM, which are located close to the putative receptor-binding reported site [33].

CDV-H protein was demonstrated to bind to hSLAM following a single mutation at position 540 [34]. Thus, it has been suggested that not only structural but also in vitro and in vivo studies for the hSLAM complexes will reveal the detailed mechanisms of these recognitions, thus explaining host specificities [26,33]. Based on the findings regarding orthologous proteins between diverse species, in addition to the closeness of humans to domesticated animals including dogs, a potential cross-species event into humans of CDV must be investigated both in silico and in vitro [11].

To assess the in vitro cross-species potential, we modelled CDV-H proteins from different strains, including those circulating in Colombia: lineage South America-3 (CDV-South-3). Canine cellular receptors were also modelled due to the absence of crystallographic structures. Molecular docking simulations were executed to find out whether changes in the amino acid sequences of the CDV-H protein from different strains imply impairments in the function of this protein in viral tropism, not only with cSLAM and canine Nectin-4 (cNectin-4) cellular receptors, but also with orthologs in humans through a computational approach. Molecular dynamics (MD) simulations were also performed, and infections of canine and human cells were carried out to evaluate whether these interactions were stable over time, trying to identify whether there is a cross-species potential of CDV into humans.

## 2. Results

### 2.1. CDV-H-South-3 Protein Diverges from the MeV-H Protein Sequence

A hierarchical analysis was carried out to establish the divergence between different CDV-H protein sequences of the strains, including CDV-H-South-3, Onderstepoort and MeV-H–2RKC (Figure 1). CDV-H-South-3 diverges in 9.9% in sequence and is in a different clade from CDV Onderstepoort H protein, which is used as a vaccine strain. On the other hand, the CDV-H-South-3 protein differs by 65.1% from 2RKC, the MeV-H protein sequence (Supplementary Table S1). The primary structure analysis suggests that CDV-H-South-3 differs from the other CDV circulating and vaccine strains. Moreover, although CDV-H protein is closely related to MeV-H protein function, there is a high divergence among both protein sequences.

### 2.2. CDV-H-South-3 Homology 3D Model and Validation

Due to the lack of crystallographic structures from either CDV or canine cellular receptors, homology modelling was employed to obtain a 3D structure of the CDV-H proteins and canine cellular receptors, which could enable evaluation of the interaction interface between the CDV-H-South-3 protein and cellular receptors. CDV-H-South-3 has an identity of 34.9% (identical residues) and 56% similarities (identity with synonymous residues changes) to 2RKC. Even though the identity was quite low, there were 397 aligned amino acids, and based on Krieger et al., it was located in the safe homology modelling zone due to the number of aligned amino acids [35]. Other modelling approaches have been used, including I-TASSER and AlphaFold2; however, for these models, where crystallographic structures of proteins with similar functions (protein from MeV) were available, the validation data favored the homology modelling (data not shown).

Figure 2A shows the template structure 2RKC and Figure 2B displays predicted models for the CDV-H-South-3 strain as a representative model.

The 3D models of the CDV-H proteins were carefully validated through computational tools, as shown in Table 1. All models located more that 95% of amino acids in favorable region for rotations and torsions by Ramachandran plot (data not shown). The overall model quality calculated with ProSA-Web indicated that all models are located within the distribution of all the proteins in the PDB that come from an X-ray crystallography (Supplementary Table S1). The TM value indicated that all models had a global folding identical to the template with values close to one (Table 1). Figure 2C shows the structural alignment between CDV-H-South-3 protein and 2RKC, exhibiting a similar overall folding. Likewise, predicted models for the canine cellular receptors were validated through the same computational approach (Table 1) obtaining quality models, with a structural alignment for human and canine SLAM, as shown in Figure 2D, illustrating a similar folding. Overall, the homology models suggest that regardless of the identities or positives between sequences, whether the function was similar, high-quality models could be obtained.

### 2.3. Molecular Docking and Dynamics between Colombian CDV-H Protein and Cellular Receptors Showed a Potential Interaction with Orthologous Human Cellular Receptors

To observe whether differences in the amino acid sequence of CDV-H protein imply changes in the affinity of derived peptides with cellular receptors, molecular docking was assessed. The docking scores obtained by AutoDock Vina for the molecular docking of different peptides from CDV-H with the cellular receptors are reported in Figure 3.

A sequence alignment of peptides shows a variation among the evaluated peptides (Supplementary Figure S1). A peptide from CDV-H-South-3 achieved a comparable docking score with the homologous peptide of MeV-H protein with hSLAM; however, when the same peptides were evaluated with cSLAM, as expected, CDV-H-South-3 had lower affinity score (−4.1 and −5.4 Kcal/mol, respectively). Regarding the Nectin-4 receptor, either from human or canine, the affinity scores were comparable with the MeV-H protein and CDV-H-South-3 peptide, corresponding to the nature of each infection. The CDV CYN07-dV strain was reported to infect non-human primates and human cell lines; the peptide derived from this strain also exhibited a high affinity score in comparison to CDV-H-South-3 with hSLAM, confirming that the Colombian strain has a greater potential to interact with human receptors in comparison with other CDV strains (Figure 3). Regarding the interaction nature, there are two changes in CDV-H-South-3 peptide in comparison with the Onderstepoort strain peptide (I542F and S546F), which could contribute to the affinity score difference. The presence of a serine instead of a phenylalanine facilitates the formation of a new hydrogen bond with the cellular receptor due to the presence of a hydroxyl group in the amino acid side chain.

To establish whether this interaction was conserved among the whole CDV-H proteins and human/canine cellular receptors, a different molecular docking tool was employed with the best affinity scores of the AutoDock Vina docking tool. The results were compared with co-crystals for both human SLAM and Nectin-4 with MeV-H protein through the interaction interface analysis. The interaction interfaces between canine SLAM and Nectin-4 were conserved, as shown in Figure 4.

The clustering results that conserved the interaction interface with MeV co-crystals are reported in Table 2, showing that all these poses are completely probable located in the clusters generated by the docking approach.

Molecular dynamics (MD) simulations were carried out to determine whether the protein–protein interaction is stable through time. MD simulation demonstrated a stable interaction in the first 15 ns with an RMSD lower than 0.3 ns, between cSLAM cellular receptor and CDV-H-South-3 protein; however, as unexpected, due to this interaction it is likely to be found in the context of natural infections of dogs with CDV, and the RMSD ranged between 0.3 and 0.5 nm until 40 ns, and then exhibited an acceptable RMSD between 0.5 and 0.65 nm, reaching 50 ns of simulation (Supplementary Figure S2A).

On the other hand, when a similar simulation was carried out with the hSLAM cellular receptor and CDV-H-South-3, after 10 ns, the simulation exhibited a lower RMSD, between 0.3 and 0.5 nm, ranging only 0.2 nm, implying a higher stability of this complex in comparison to the cSLAM cellular receptor and CDV-H-South-3 protein, which, in fact, suggests a potential interaction between the hSLAM cellular receptor and CDV-H-South-3 (Supplementary Figure S2B).We therefore concluded that MD simulation of hSLAM cellular receptor and CDV-H-South-3 protein demonstrates the reliability of the in silico approach regarding the molecular docking of either CDV-H protein or human cellular receptors in comparison to crystallographic statures of the MeV interaction complex with human receptors elucidated from the infection context. Although the cSLAM cellular receptor and CDV-H-South-3 protein complex are characterized in natural infections, this complex exhibited an interaction interface less stable than the hSLAM cellular receptor and CDV-H-South-3 protein complex, from the molecular dynamic’s perspective.

### 2.4. CDV from Colombian Circulating Strain Was Isolated from a Viremic Patient

Nasal swab samples were filtered from a PCR-positive serum patient and reference CDV from Nobivac vaccine. Virus isolations were performed in Vero-Dog-SLAM cells and the presence of CDV was confirmed by titration and qPCR. Both isolates were stored at −80 °C until cell line infection assays and protein expression detection.

### 2.5. CDV Proteins from Colombian Isolate Was Immunodetected in Cell Monolayers by Monoclonal Antibodies

The viral titer was 2.5 × 10^8^ PFU/mL for the wild-type CDV isolated from a viremic patient and 1.5 × 10^5^ PFU/mL for the reference CDV strain. To determine whether there was a difference in protein expression from CDV Colombian strain compared to a reference isolate (Onderstepoort) from a modified live vaccine, detection by monoclonal antibodies by immunoblotting and CELL-ELISA was performed. As shown in Figure 5A, Vero-dog-SLAM cell lysates contained a greater amount of CDV protein when infected at the same MOI by the wild-type strain, compared to the reference strain (Onderstepoort). This finding was observed by both Western blot and CELL-ELISA (Figure 5A,B). CDV proteins were not detected in the supernatants for either virus, exhibiting a differentiated protein expression pattern in comparison to the reference CDV.

### 2.6. CDV Colombian Strain Could Infect Human Cell Lines Efficiently

To confirm the in silico results suggesting that CDV-H-South-3 can infect human cell lines, an in vitro study was performed using both human and canine cell lines infected with the wild-type and the reference Onderstepoort strains. The monocytic cell line U937, was highly permissive to the reference CDV strain, and comparable to the Vero-Dog-SLAM. Furthermore, both A549 and MCF-7 exhibited lower viral titers, as shown in Figure 6. On the other hand, when the wild-type CDV strain was employed for cell infection, MCF-7, a breast adenocarcinoma cell line, which likely expresses hNectin-4, had a higher viral titer than the other cell lines. After molecular detection through the qPCR of CDV in the infected monolayer, the obtained results were consistent with the plaque assay infectious viral particles measurement, indicating a replicative process of either reference or wild-type CDV strains. Notbaly, the canine MDCK cell line was not infected with either reference or wild-type CDV strains (Figure 6). As expected, the reference CDV isolate was adapted to cell lines, enabling the employment of any cellular receptor to infect a susceptible cell line monolayer. However, when the wild-type CDV strain was evaluated, the results were on the same line to what was reported elsewhere regarding wild-type CDV strain’s capacity to use hNectin-4 as a cellular receptor, in the MCF-7 cell line; however, either way, it could infect U937 with less effectivity.

## 3. Discussion

CDV is a pathogen that affects a vast array of animal species, including domestic dogs, wild animals and non-human primates [2]. However, to date, the potential cross-species transmission to humans has not been fully understood [36,37,38]. Considering CDV as potential zoonotic virus has important implications in public health, due to the proximity among potential transmitters such as domestic dogs and humans. Hence, more studies are crucial to identify the key molecular aspects that could mediate this event.

For *Morbilliviruses*, the interaction between H protein and its cellular receptors is highly specific depending on certain amino acids. Changes in the binding domain could result in abortive protein–protein interactions; therefore, amino acid changes could result in a failure of virus attachment to cellular receptors [6]. In this study, a hierarchical analysis was developed to compare diverse H glycoprotein sequences by a protein phylogenetic construction. As expected, CDV-H-South-3 differed from both MeV and reference CDV-H protein (Figure 1), which could imply an impairment of the function of this protein in viral tropism [12]. Despite identification of the interaction interface between both hSLAM and hNectin-4 with MeV-H protein, as well as the specific amino acids involved being reported [29], there are a lack of experimental data on crystallographic structures to study this phenomenon in CDV.

Homology modelling is a helpful approach to understand information at the molecular level of proteins, because the difference in the number of reported sequences in databases is lower than the crystallographic structures in PDB [39]. Similar structures and functions have been shown for viruses within homologous families, without the need for high amino acid identity between the sequences [40]. We have used homology modelling to construct models of not only the CDV-H-South-3 based on MeV-H protein, but also canine SLAM and Nectin-4 cellular receptors based on amino acid sequences reported in the NCBI (Figure 2). Regardless of the low identity between MeV and CDV-H proteins, MeV-H can still be considered a suitable template structure for CDV-H modelling, because after validation, CDV-H-South-3 model was a reliable structure (Table 1). This could be due to the equivalent function of the H proteins in their respective viruses.

Although receptor usage has been considered as a main aspect in *Morbillivirus* cross-species transmission, because CDV has been demonstrated to be a pathogen with a wide range of susceptible animal species, its cross-species transmission potential is proposed to be multifactorial due to the high promiscuity of CDV. Therefore, orthologous receptors in other species with high homology will not imply host specificity in morbilliviruses, as has been demonstrated in CDV transmission dynamics [13,38]. CDV has a negative, single-stranded RNA genome; thus, acquiring changes in the receptor-binding regions of H protein for better adaptation to diverse host species has commonly been reported. Moreover, because the role of those mutations is not completely elucidated, they must contribute to the expanding generalist host-range of CDV via different receptor-specific interactions [41]. However, considering that CDV could jump to other species as a generalist agent and become a specialist in certain species [13], CDV has the potential to infect other species, including humans, without a long genomic change requirement, as shown in the in silico and in vitro approach of the present study.

The cross-species transmission potential of CDV to humans has been proposed prior to this study [36,37,42,43]. The CDV Ac96I strain was reported to infect human epithelial cell lines expressing the Nectin-4 cellular receptor, but not hSLAM [44]. On the other hand, it has been reported that the recombinant wild-type CDV-A75/17 infected Vero cell lines modified to express the hSLAM cellular receptor [34]. Other studies have suggested that the codon usage of CDV is more related to human codon usage bias (CUB) instead of the canine CUB, probably because the virus or its progenitor was initially adapted to humans [45]. Finally, the CDV CYN07-dV strain was isolated from non-human primates, which could employ macaque cellular receptors as efficient canine cellular receptors, providing evidence of the capacity of CDV to jump to non-human primates [46]. Moreover, it has also been reported that the CDV-H protein could interact with the N-terminal region of macaque SLAM in a stable form through specific mutations, due to a single mutation in residue 28 (histidine instead of arginine) which could destabilize the interaction. On the other hand, methionine in residue 29 of MeV-H protein has exhibited a stabilizing capacity between hSLAM and MeV-H protein, indicating the importance of recognizing specific amino acids in CDV-H protein that could enable the cross-species transmission of CDV into humans [47,48].

As shown in Figure 3, CDV-H-South-3 exhibited a favorable affinity score when docked by AutoDock Vina with both human and canine cellular receptors (−5.4 and −5.3 Kcal/mol, respectively), especially SLAM cellular receptor, in comparison to the MeV-H protein (−5.1 Kcal/mol). Additionally, as reported in vitro previously with other CDV strains [34], our findings suggest that the CDV-H-South-3 protein could interact with human receptors, delineating the potential cross-species transmission in silico, explained by the capacity of the CDV-H-South-3 protein to interact with human receptors. Additionally, as shown in Supplementary Figure S1, the presence of a serine in CDV-H-South-3 enables the formation of a new hydrogen bond, implying a lower affinity score with the SLAM receptor. There was also a difference of the Onderstepoort strain and CDV-H-South-3 score when assessed with hSLAM, suggesting that vaccine strains have differences not only in amino acids sequences, but also in the interaction of this strain with cellular receptors [20]. The importance of this result is supported by a well-known aspect of CDV infection, where the SLAM cellular receptor is crucial for the initial steps of CDV pathogenesis [5]. However, regardless of the high identity among human and canine Nectin-4 and other studies which have reported that CDV-infected cell lines express hNectin-4, there are no favorable affinities with CDV-H-South-3, indicating a probable specificity among strains for the usage of different cellular receptors. Co-crystallographic structures come from the context of the infection; therefore, comparison among them and the complexes obtained through computational approaches enable demonstration of the importance of a conserved interaction interface between viral H protein and cellular receptors [29,30].

Using the molecular docking tool ClusPro (Figure 4 and Table 2), it was possible to demonstrate that the interaction interface of cSLAM and cNectin-4 with CDV-H-South-3 is conserved when compared to a co-crystallographic structure between hSLAM or hNectin-4 and MeV-H protein (Figure 4) (PDB CODE: 3ALX and 4GJT), indicating the quality and reliability of the in silico approach. When hSLAM or hNectin-4 were docked with CDV-H-South-3, even though the interface is not completely identical, the CDV-H interaction peptide with cellular receptors remains at the same interface as shown in the co-crystal [29,30], although there are some variations in the amino acid sequence, as shown in Supplementary Figure S1. Moreover, our models suggest an interaction between CDV-H protein and the SLAM cellular receptor (Figure 4), in comparison to the co-crystal of MeV-H protein and its receptor. Despite three amino acid changes between MeV and CDV-H protein, it is important to highlight the similarity of human and canine cellular receptors, which has been reported as higher than 94% with hNectin-4 and less than 80% with hSLAM [49].

In this study, molecular dynamics simulations were carried out to establish whether complexes obtained by molecular docking are stable through time, as well as having favorable affinity scores. [50]. Multiscale molecular dynamics simulations have been performed to construct a mechanistic understanding of viral pathogens regarding the structure and their dynamics, with simulations times around 10–13 ns [51]. Here, we carried out 50 ns simulations, either with cSLAM or hSLAM cellular receptors and the CDV-H-South-3 interaction peptide, as exhibited in Supplementary Figure S2, in an attempt to recognize different aspects of the viral tropism as viral protein and cellular receptor interactions. With an RMDS lower than 0.3 nm among all trajectory poses found through the simulation time, this suggests a stable complex between the hSLAM cellular receptor and CDV-H-South-3 interaction peptide. For other viral models such as the influenza A virus (IAV), H5N1, MD simulations with times of 15 ns have been employed to elucidate the effects of single mutations in the H protein in the host [52], and MD studies of virus–host receptor complexes have been conducted to compare the contributions of water in these interactions [53].

Considering our in silico predictions, a CDV in vitro model was employed to evaluate whether the CDV-South-3 isolate could infect human cell lines in comparison to the reference strain. Hence, the Colombian CDV isolate has the capacity to infect human cell lines efficiently in vitro in a low multiplicity of infection (MOI = 0.1), likely employing the hNectin-4 cellular receptor in an epithelial cell line and a monocytic cell line which expresses hSLAM. Additionally, to evaluate whether there were differences in protein expression between them, CELL-ELISA and Western blotting was carried out, demonstrating a higher protein expression from CDV-South-3 compared to the reference strain (Figure 5). This may imply differences in the infectivity and CDV-H protein interaction with cellular receptors between both isolates, enabling determination of a specific protein expression profile [54].

Specific mutations on CDV-H have been demonstrated to enable CDV developing the ability to infect human cell lines. In cells expressing hSLAM that were infected with CDV, syncytia formation was observed, and when substitutions of the protein H were studied, it was found that a single amino acid change allowed the CDV-H protein to employ the hSLAM receptor, suggesting that, at least at the receptor level, humans could be susceptible to CDV infection [32,33,44]. In this study, we have demonstrated, from an in silico and in vitro approach, that both a reference and a Colombian CDV isolate could interact with human cellular receptors and infect human cell lines efficiently (Figure 3, Figure 4 and Figure 6). Notably, CDV can encounter resident dendritic cells and alveolar macrophages of the respiratory tract, which become infected through the SLAM receptor. These infected cells transport CDV to the lymph nodes, where activated T and B cells are also infected using the SLAM receptor, resulting in the amplification of the virus and the onset of primary viremia [6,11]. It has been proposed that CDV evolution and dynamics could lead to the emergence of CDV variants, because of adaptations that play a different role in the virus transmission, viral tropism, species susceptibility and virulence. The substitutions of D540G and M548T in the H protein, Y267C in the V protein, C116Y in the F protein, and M267V in the phosphoprotein have enabled cell infection in human H358 cells [26]. Thus, whether CDV-H protein could interact with hSLAM, and the important changes required for this, has become a key research aspect to elucidate the potential cross-species transmission of CDV into humans due to its important role in viral tropism.

Dogs and non-human primates vaccinated with an MeV vaccine have exhibited activation of the immune response with cross-reactive activity to CDV even in the presence of maternal antibodies [55,56]. This leads us to wonder whether CDV could jump the species barrier to infect humans and cause a clinical disease, as has been already described in non-human primates [31,46,57]. In MeV-vaccinated and CDV-infected cynomolgus macaques, MeV-specific neutralizing antibody levels were boosted by CDV challenge infection, suggesting that cross-reactive neutralizing epitopes exist and that cross-reactive cellular immune responses were also present [42]. This might be due to the presence of conserved epitopes between MeV and CDV-H proteins, which are around 36% identical, and in the protein function. Considering that the host range of CDV is not completely understood, in terms of the main aspects that enable CDV to overwhelm a vast array of animal species, the modulation of the innate immune response could play an important role because it has been demonstrated that some morbilliviruses, such as MeV, can modulate the immune response basically depending on the species, via the V protein and virus type. Hence, those facts could explain how CDV could not affect different animals based on the capacity to counteract innate immunity in the host [38,49]. In the scenario in which MeV is eradicated from an area and vaccination for this virus becomes unnecessary, it could be possible to determine whether immunity against MeV has been protecting humans against CDV infection, or at least the presentation of clinical signs [34,44].

## 4. Materials and Methods

### 4.1. H Protein Primary Structure Analysis, Homology Modelling and Models Validation

The sequences of the H glycoprotein of the wild-type and vaccine CDV strains were downloaded from GenBank (https://www.ncbi.nlm.nih.gov/nucleotide/, accessed on 1 January 2021), with accession numbers: AAG15490.1 (Onderstepoort used as CDV reference strain), KF835413.1 (CDV-H-South-3 strain). In addition, the canine cellular receptors: AAK97460 (canine SLAM), AGB56848 (canine Nectin-4) were retrieved from the same database. A hierarchical analysis was used to compare diverse H glycoprotein sequences by phylogenetic construction using MEGA7.0 [58]. Briefly, a multiple sequence alignment was built; then, the substitution model was calculated for the dataset and the model with the lowest Bayesian Information Criterion score was considered to describe the substitution pattern. Consequently, the molecular phylogenetic analysis was inferred by using a maximum likelihood method, based on a JTT matrix-based model [59]. An initial tree for the heuristic search was obtained by applying the neighbor-joining method to a matrix of pairwise distances estimated using a JTT model. A discrete gamma distribution was used to model evolutionary rate differences among sites. The analysis involved 40 protein sequences. Homology models were constructed to study the interaction of viral proteins and cellular receptors. The amino acid sequence of the CDV-H from the SouthAmerica-3 lineage strain (CDV-H-South-3), CYN07-dV (accession number AB687720), an isolate from non-human primates and Onderstepoort strain, were obtained from the NCBI. To obtain a homologous template, a BLASTP search was carried out using each protein against the PDB database. The templates for modelling the canine cellular receptors were search directly in PDB. The hSLAM protein complexed with the MeV (3ALX) was used as a template for modelling the cSLAM protein and the hNectin-4 (4GJT) receptor was used to model the cNectin-4. MODELLER v. 9.22 was used to model the 3D structure of the CDV-H ligand and the canine receptor proteins. After running the program, 100 different structures with model quality scores (molpdf, DOPE, GA341) [60] were obtained. The generated homology models and the respective templates were overlapped to establish the root mean square deviation (RMSD) differences between the model and template structures utilizing TM-Align, a protein structure alignment algorithm based on the TM-score [61]. The homology models were assessed using the bioinformatics tools SWISS-MODEL™, which provides global and local model quality based on the Z-score and QMEAN, in addition to each residue quality calculation from the amino acid sequence [62]. ProSA-Web, another Z-score for the overall model quality, was used to check whether the Z-score value of the input structure was within the range of scores typically found for native proteins of similar size, with PDB as the reference database [63]. The Ramachandran plots (RAMPAGE) were calculated to establish amino acids in energetically favorable regions, regarding dihedral angles ψ against φ of amino acid residues in protein structure [64].

### 4.2. Molecular Docking Analysis

CDV-H protein and host cellular receptor interactions were assayed by employing two molecular docking online tools, AutoDock Vina [65] and ClusPro online tool [66,67] (accessed on 1 April 2021). Docking evaluation was performed with both canine and human cellular receptors. For AutoDock Vina analysis, a 25 amino acid domain from either CDV-H protein or MeV-H protein were extracted and denominated as the flexible ligands. The crystallographic structure of MeV-H protein and its cellular receptors enable selection of the interaction interface and were used to delimitate the docking box with a spacing of 1 Å and 50 xyz points, with centers defined for each complex and with an exhaustiveness of 10. Polar hydrogens and Gasteiger charges were added to the ligand with AutoDock Tools from MGL Tools (accessed on 1 April 2021). The affinity between the 25-amino acid ligand and host cellular receptors was determined based on binding energy in Kcal/mol over three runs with AutoDock Vina and the RMSD value. For ClusPro examination, the complete CDV-H protein and the four domains from the CDV-H protein were docked to the host cellular receptors. For this analysis, both the ligand and the receptor were considered rigid structures. The most probable pose was selected based on the tool scores. Graphic analyses of all 3D complexes generated were performed using the software PyMOL, Molecular Graphics System, Version 2.0 (Schrödinger, LLC, New York, NY, USA).

### 4.3. Molecular Dynamics Simulations

Molecular dynamics simulations were performed using GROMACs 5.1.521. We evaluated the complexes of canine and human SLAM and the CDV-H-South-3 interaction peptide. The topology of the protein was generated with AMBER99SB19; the protein–peptide complexes were solvated with TIP3P explicit water molecules and places in the center of a dodecahedron with minimum of 1 Å distances maintained between the complex and the edge of the box. The charge of the system was neutralized by adding ions of Cl and Na. The steepest descent approach through 50,000 steps was performed for each complex for energy minimization. Two parameters were evaluated for energy minimization: first, that the potential energy was negative; and second, that the maximum force, Fmax, was no greater than 1000 KJ mol^−1^ nm^−1^. NVT with the V-rescale and NPT with Parrinello–Rahman was performed for 100 picoseconds, to equilibrate the system for a constant volume, pressure (1.05 bar) and temperature (300 K). The final molecular dynamics simulation was run for 50 ns for each complex and the trajectories were used for analysis with Xmgrace software (Oregon Graduate Institute of Science and Technology, Hillsboro, OR, USA).

### 4.4. Cell Lines, Virus Isolation, and Viral Titration

Vero cells line expressing dog signaling lymphocyte activation molecules (named Vero-Dog-SLAM) were used to isolate, replicate, and titrate reference and wild-type CDV (kindly donated by Yusuke Yanagi from Kyushu University, Fukuoka, Japan). For cell line assays, human cell lines of A459 (human lung adenocarcinoma), MCF-7 (human breast adenocarcinoma) expressing hNectin-4, U937 (human histiocytic lymphoma) expressing hSLAM and canine cell line as MDCK (Madin–Darby canine kidney) from the ATCC were employed and cultured in Dulbecco’s modified Eagle’s medium (DMEM) supplemented with 2% fetal bovine serum (FBS) (Gibco, Grand Island, NY, USA) and 1% antibiotic/antifungal at 37 °C in a humidified atmosphere containing 5% CO_2_. Wild-type and reference virus isolation was carried out from a symptomatic dog from Medellin, Colombia [26], and CDV Nobivac vaccine (MSD Animal Health, Summit, NJ, USA), respectively, following the same procedure. The Colombian viral isolate is the subject of a contract for access to genetic resources and derived products No. 132 of 2016 RGE0177, signed with the Ministry of Environment and Sustainable Development of the Republic of Colombia. Briefly, nasal swabs or vaccine solution were filtered and inoculated for 2 h at 37 °C to allow virus adsorption, with shaking every 15 min for uniform virus distribution in 6-well plates of Vero-Dog-SLAM monolayers with 500 μL inoculum. The inoculum was not removed, DMEM was supplemented with 2% FBS to complete 1.5 mL, and infection was continued until the characterized cytopathic effect was identify. Viral titration was performed in Vero-Dog-SLAM cells (1.5 × 10^5^) seeded into 24-well plate and inoculated with serial dilutions of supernatants. After a 2 h incubation, the viral inoculum was removed and washed twice with phosphate-buffered saline (PBS). Then, solid DMEM with 0.4% of agarose was supplemented with 2% FBS. The plaque formation continued for 3–5 days, and monolayers were fixed using 4% formaldehyde and stained with crystal violet for plaque counting.

### 4.5. Molecular Detection of Wild-Type Colombian CDV Strain by RT-PCR

To assess the molecular CDV detection, total RNA was extracted from either supernatants or field samples using QIAamp Viral RNA Mini Kit (QIAGEN^®^, Hilden, Germany), in accordance with the manufacturer’s instructions. Reverse transcription was carried out with the High-Capacity cDNA Reverse Transcription Kit (Thermo Scientific^®^, Waltham, MA, USA). Viral cDNA was detected using morbillivirus universal primers (forward: 5′-ATGTTTATGATCACAGCGCGGT-3′ and reverse: 5′-ATTGGGTTGCACCACTTGTC-3′) with the genomic position 2132–2541 for amplifying a 429 bp fragment of the phosphoprotein gene [68]. Real-time PCR was performed with the Power Up™ SYBR Green Master Mix kit (Thermo Scientific^®^), following the manufacturers’ instructions, with the following thermal conditions: initial denaturation at 95 °C for 4 min followed by 35 cycles of denaturation at 95 °C for 30 s, annealing at 50.8 °C for 30 s, and extension at 72 °C for 1 min. Ultrapure water was used as a negative control and cDNA from one of the vaccines was the positive control. Samples were amplified in a QuantStudio3 thermocycler (Thermo Scientific^®^).

### 4.6. CDV Protein Detection by CELL-ELISA and Western Blot

For CELL-ELISA, Vero-Dog-SLAM cell monolayers were infected with either reference or wild-type CDV. Non-infected cells were employed as controls. All were fixed with 4% PFA and treated with 0.1% Triton X-100. Then, 0.3% H_2_O_2_ with 10% methanol in PBS was added; subsequently, non-specific antibody binding sites were blocked with 10% BFS-PBS. Infected and non-infected cells were incubated at 4 °C with anti-H-CDV protein (Invitrogen^®^, Thermo Scientific^®^) G34B mouse monoclonal antibody overnight at 1:200 concentrations. Subsequently, they were incubated with an anti-mouse-HRP secondary antibody for 30 min at room temperature. Finally, 3,3′,5,5′-tetramethylbenzidine (TMB; Invitrogen^®^, Carlsbad, CA, USA) was added. The absorbance was read at 620 nm using a Multiskan™ FC Microplate Photometer (Thermo Scientific^®^) reader. For immunoblots, Vero-Dog-SLAM cells were infected with either reference or wild-type CDV at the multiplicity of infection (MOI = 0.1) and incubated for 72 h at 37 °C in 5% CO_2_. Uninfected cells were negative controls. Radioimmunoprecipitation assay buffer (RIPA buffer) was employed to extract proteins from either infected or uninfected cell monolayers. The total protein amount was quantified with Bradford assay (Sigma Aldrich^®,^ St Louis, MO, USA) with a standard curve with bovine serum albumin (BSA). Amounts of 40 milligrams from each condition were submitted to sodium dodecyl sulfate polyacrylamide gel electrophoresis (SDS-PAGE) with 5% stacking gel and 10% separating gel. Separated proteins were transferred to a PVDF membrane at constant electricity (25 mV, overnight). Subsequently, the membrane was blocked with BSA in TBST for 2 h at room temperature. Afterwards, the membrane was incubated with anti-H-CDV protein (Invitrogen^®^) DV2-12 mouse monoclonal antibody overnight and anti-β-actin rabbit monoclonal antibody for constitutive gen, then washed three times with TBST, and incubated with a 1:2000 dilution of horseradish peroxidase (HRP)-conjugated goat anti-mouse IgG (BioRad^®^, Laboratories, Hercules, CA, USA) for 1 h at room temperature. The Clarity Western ECL Substrate was employed, and finally, the blots were analyzed with G: BOX Chemi XRQ by chemiluminescence.

### 4.7. Reference and Wild-Type Colombian CDV Strain Infection in Human and Canine Cell Lines

Cell monolayers from either human or canine cell lines were infected. Briefly, cell lines were harvested and seeded in 24-well plates and inoculated after 24 h. Cells were infected with MOI = 0.1, and after 2 h incubation, the viral inoculum was removed and washed twice with phosphate-buffered saline (PBS). Then, DMEM supplemented with 2% FBS (Gibco, Grand Island, NY, USA) was added, and infection was followed for 72 to 96 h. Two independent experiments with 3 replicates (*n* = 6) were carried out in each cell line, and non-infected cells were employed as negative controls. Molecular detection was conducted in infected monolayers. Supernatants were evaluated for infectious viral particles by plaque formation assays, reporting the viral titer. Means and standard deviations were reported.

## 5. Conclusions

We have elucidated that CDV-South-3, circulating in Colombia, has the potential to infect human cell lines by interacting with orthologous human receptors, at least from an in silico and in vitro approach, suggesting the potential cross-species transmission of CDV to humans. In vivo research must be performed to understand all the main aspects that imply the transmission potential. Based on the current proximity of dogs to humans, the cross-species transmission could be a constant threat. Additional evidence that this could be possible includes infections in non-human primates and the cross-neutralization capacity of MeV antibodies to CDV, employing the same animal model. Altogether, this study suggests that there should be a priority to prove whether this hypothesis is viable in nature: MeV eradication is a World Health Organization goal, and if achieved, cessation of vaccination for MeV may allow another morbillivirus, such as CDV, to take over this ecological niche.

## Figures and Tables

**Figure 1:** Hierarchical analysis of CVD-H amino acid sequences from diverse strains, including MeV-H protein sequence. The phylogenetic tree was inferred by the maximum likelihood method using a bootstrap of 1000. All the GenBank accession numbers and the viral protein are shown in all branches. Numbers on the nodes are the bootstrapping values for each clade. The CDV-H-South-3, Onderstepoort strain and MeV-H protein sequences are shown with a black filled circle, black filled diamond, and black filled square, respectively.

**Figure 2:** Homology models obtained by Modeller^®^ and structural alignment with template. (**A**) The MeV-H protein used as template. PDB CODE: 2RKC. (**B**) Homology model of CDV-H-South-3 protein. (**C**) Structural alignment of 2RKC template (green) and CDV-H-South-3 protein model (light blue). (**D**) Structural alignment of hSLAM (green) and the cSLAM model (orange) as an example of modeled anine receptors.

**Figure 3:** Score values of the molecular docking by AutoDock Vina of peptides from different MeV or CDV strains.

**Figure 4:** Structural alignment from co-crystals of CDV-H or MeV-H protein with either human or canine SLAM and Nectin-4. Structural alignments between (**A**) the co-crystal of hSLAM (blue) and MeV-H protein (cyan) downloaded from the PDB (PDB Code: 3ALX) and the complex of cSLAM (orange) and CDV-H-South-3 (green) obtained by ClusPro and (**B**) the co-crystal of hNectin-4 (blue) and MeV-H protein (cyan) downloaded from the PDB (PDB Code: 4GJT) and the complex of cNectin-4 (orange) and CDV-H-South-3 (green) obtained by ClusPro.

**Figure 5:** CDV protein immunodetection using monoclonal antibodies in CELL-ELISA and immunoblotting. (**A**) Western blotting reference and wild-type CDV strains. Supernatants and Vero-Dog-SLAM cell lysates were submitted to 10% SDS-PAGE gels and analyzed with monoclonal antibodies to detect CDV proteins. Actin was measured as a constitutive gene, positive for cell lysates; Molecular Weight, MW; reference CDV supernatant, 1; Vero-Dog-SLAM cell lysates (negative control), 2; wild-type CDV supernatant, 3; reference CDV infected Vero-Dog-SLAM cell lysates, 4; wild-type CDV infected Vero-Dog-SLAM cell lysates, 5. (**B**) CELL-ELISA for CDV protein detection in reference and wild-type CDV strains.

**Figure 6:** Reference and wild-type CDV infection in both human and canine cell lines. U937, A549 and MCF-7 human cell lines and MDCK canine cell lines were infected with either reference or wild-type CDV. Vero-Dog-SLAM was employed as a positive control. Experiments on each cell line were performed by two independent experimental units with three replicas each (*n* = 6). Non-infected cells were employed as negative controls. Means and standard deviations are shown in the bar graph.

**Table 1:** Validation data of all models obtained by homology modelling.

Protein	Z Value	Favorable Region (%)	TM Value	Aligned AA
CDV-H-South-3	−7.00	96.9	0.983	397
CYN07-dV	−6.82	98.1	0.986	399
Onderstepoort	−6.53	97.2	0.985	397
cSLAM	−4.56	97.2	0.992	104
cNectin-4	−4.55	98.2	0.998	114

**Table 2:** Clustering analysis of molecular docking by ClusPro approach.

Complex	Cluster	Members
cSLAM–CDV-H-South-3	2	49
hSLAM–CDV-H- South-3	6	32
cNectin-4–CDV-H- South-3	3	54
hNectin-4–CDV-H- South-3	4	37

## Data Availability

Not applicable.

## Supplementary Materials

The following are available online at https://www.mdpi.com/2076-0817/10/9/1199/s1, Figure S1: Interaction domain of either MeV or CDV-H protein; Figure S2: Interaction domain of either MeV or CDV-H protein; Table S1: Identity percentage of modelled proteins and employed templates with PDB number.
